# Responses of Rapid Viscoanalyzer Profile and Other Rice Grain Qualities to Exogenously Applied Plant Growth Regulators under High Day and High Night Temperatures

**DOI:** 10.1371/journal.pone.0159590

**Published:** 2016-07-29

**Authors:** Shah Fahad, Saddam Hussain, Shah Saud, Shah Hassan, Bhagirath Singh Chauhan, Fahad Khan, Muhammad Zahid Ihsan, Abid Ullah, Chao Wu, Ali Ahsan Bajwa, Hesham Alharby, Amanullah, Wajid Nasim, Babar Shahzad, Mohsin Tanveer, Jianliang Huang

**Affiliations:** 1 National Key Laboratory of Crop Genetic Improvement, MOA Key Laboratory of Crop Ecophysiology and Farming System, College of Plant Science and Technology, Huazhong Agricultural University, Wuhan, Hubei, 430070, China; 2 College of Resources and Environment, Huazhong Agricultural University, Wuhan, Hubei, 430070, China; 3 Department of Horticulture, Northeast Agricultural University, Harbin, 150030, China; 4 Department of Extension, Agricultural University Peshawar, 25130, Khyber Pakhtunkhwa, Pakistan; 5 Queensland Alliance for Agriculture and Food Innovation (QAAFI), The University of Queensland, Toowoomba, 4350, Queensland, Australia; 6 Department of Arid Land Agriculture, Faculty of Meteorology, Environment & Arid Land Agriculture, King Abdul Aziz University P.O. Box 80208, Jeddah, 21589, Saudi Arabia; 7 School of Agriculture and Food Sciences, The University of Queensland, Gatton, Queensland, 4343, Australia; 8 Department of Biological Sciences, Faculty of Science, King Abdulaziz University, 21589, Jeddah, Saudi Arabia; 9 Department of Agronomy, Faculty of Crop Production Sciences The University of Agriculture, Peshawar, 25000, Pakistan; 10 Department of Environmental Sciences, COMSATS Institute of Information Technology (CIIT), Vehari, 61100, Pakistan; 11 Agricultural University, Faisalabad, 38000, Pakistan; 12 Hubei Collaborative Innovation Center for Grain Industry, Yangtze University, Hubei, China; Clemson University, UNITED STATES

## Abstract

High-temperature stress degrades the grain quality of rice; nevertheless, the exogenous application of plant growth regulators (PGRs) might alleviate the negative effects of high temperatures. In the present study, we investigated the responses of rice grain quality to exogenously applied PGRs under high day temperatures (HDT) and high night temperatures (HNT) under controlled conditions. Four different combinations of ascorbic acid (Vc), alpha-tocopherol (Ve), brassinosteroids (Br), methyl jasmonates (MeJA) and triazoles (Tr) were exogenously applied to two rice cultivars (IR-64 and Huanghuazhan) prior to the high-temperature treatment. A Nothing applied Control (NAC) was included for comparison. The results demonstrated that high-temperature stress was detrimental for grain appearance and milling qualities and that both HDT and HNT reduced the grain length, grain width, grain area, head rice percentage and milled rice percentage but increased the chalkiness percentage and percent area of endosperm chalkiness in both cultivars compared with ambient temperature (AT). Significantly higher grain breakdown, set back, consistence viscosity and gelatinization temperature, and significantly lower peak, trough and final viscosities were observed under high-temperature stress compared with AT. Thus, HNT was more devastating for grain quality than HDT. The exogenous application of PGRs ameliorated the adverse effects of high temperature in both rice cultivars, and Vc+Ve+MejA+Br was the best combination for both cultivars under high temperature stress.

## Introduction

Global agriculture has reached a time of crisis. In this coming century, drastic changes in agriculture systems are expected, and the main driving force for these changes will be global warming [1]. The harshness of warmer climates has already been observed in terms of the recurrent incidence of heat stress, and these changes have severely reduced the quality and yield attributes of susceptible crops such as rice. To cope with these changes and identify suitable rice cultivars and different mechanisms to achieve better performance under these conditions requires much effort from the scientific community. Since 1960, a 1.2°C enhancement in the mean temperature has been recorded in China [2]. Because considerable spatiotemporal and seasonal unpredictability have been associated with the warming tendency [3], agriculture acclimatization against these climate alterations and advanced research are needed both on the spatial scale and regionally [4]. Globally crop production is facing a challenging task from mounting temperatures [5]. An increase of 1°C daily mean minimum temperature for a growing season may lead to a 10% grain yield loss of rice [6]. Similar estimates for wheat showed a reduction of 3–4% in yield for every 1°C increase in temperature above 15°C [7], and declines of 1% in maize yield occur for every day spent above 30°C [8].

Heat stress is defined as an increase in temperature beyond a threshold level for a period of time that is sufficiently long to cause irreversible harm to plant growth and development. Nevertheless, heat stress is a multifaceted function of intensity (temperature in degrees), duration, and rate of temperature increase. A potential threat to rice production and sustainability has been observed because of the augmented occurrence and potency of high temperature, together with high unpredictability. Rice is an important and staple food crop for approximately half of the world’s population. It supplies 52–76% of the total calories consumed in the diets of individuals in countries such as Bangladesh, Cambodia, Indonesia, Myanmar and Vietnam and 30% of the calories consumed by Indian and Chinese populations [9]. For several years, rice has been utilized as a model plant, but studies concerning high day and night temperate stress are needed to boost the growth attributes of this crop [10]. By the end of the 21^st^ Century, rice yields are estimated to be reduced by 41% [11]. Rice is more susceptible to high temperatures at the flowering stage than it is at the vegetative stage; thus, the reproductive stage is severely affected by high temperatures [12, 13].

Rice quality traits include milling, physical appearance, nutritional value and cooking and eating [14]. The assessment criteria for milling quality generally include brown rice percentage, milled rice percentage and head rice percentage, which reflects the proportion of entire kernels (head rice or head milled rice) and broken kernels that are produced during the milling of rough rice. These criteria are closely associated with the market value because broken milled rice is less than half of the price of head milled rice [15]. The appearance quality of rice is primarily determined by the grain size, translucency, chalky grain percentage, chalky area and chalky degree. Chalky grains have opaque spots in the endosperm that range in size, either on the dorsal side of the grain (white belly) or in the center (white center) [16]. Cooking and eating qualities are primarily specified based on the amylase content, gelatinization temperature, and starch gel consistency [17]

During kernel development, environmental temperature plays a fundamental part in generating unexpected variations in rice grain quality [18]. For example, high night temperature (HNT) affects kernel development and significantly reduces head rice yield [19]. Similarly, increased chalkiness formation [20], reduced amylose content and smaller grain size [18, 21] were observed in the high-temperature stress grains. Moreover, flour and bread characteristics and other physico-chemical attributes of grain crops [22], including variations in flour protein ingredient [23] during the grain filling stage, can vary due to high temperatures. Exposure of HNT during grain filling stage altered the enzymatic activity [18, 24], leading to irregular packing of starch granules resulting in the increased chalkiness [25]. Nevertheless, changes in the grain shape and cooking quality under high temperature are still poorly understood. Recently, Shi et al. [26] reported that HNT reduced in head rice yield and grain width, altered the amylose content, while increased the increased the chalkiness in various studied genotypes. The adequate utilization of the genotypic alterations in rice [27] and the use of different chemical applications and precise combinations could improve the rice performance against mounting temperatures. However, due to the scarce literature on these two mechanisms, studies concerning the potential effects of these strategies on the qualitative traits of rice are needed.

The ascorbic acid (vitamin C; Vc), alpha-tocopherol (vitamin E; Ve), brassinosteroids (Br), methyl jasmonates (MeJA), and triazoles (Tr) that were utilized in this experiment are pivotal in enhancing the agronomical and physiological attributes associated with thermoresistance [28, 29, 30, 31]. Ascorbate (vitamin C) occurs in all plant tissues, with higher concentrations in photosynthetic cells and meristems. Approximately 30 to 40% of the total ascorbate is present in the chloroplast, and stromal concentrations as high as 50 mM have been reported [32]. Ascorbic acid (AsA) is a significant antioxidant that reacts not only with H_2_O_2_ but also with O^−^_2,_ OH and the lipid hydroperoxidases produced from aerobic metabolic processes, such as photosynthesis and respiration, or in response to environmental stresses, such as heat, drought, cold, and pollutants [33, 34]. AsA is water soluble and has a supplementary function in defending or reviving oxidized carotenoids or tocopherols [34]. Vitamin E (α-Tocopherol) is present in green parts of plants. Through the concerted action of other antioxidants, this compound scavenges lipid peroxy radicals [35, 36]. Further, tocopherols were also recognized as physical quenchers and chemicals that react with O_2_ in chloroplasts to defend the PSII structure and function [37, 38]. In turf grass, a two-fold increase in α-tocopherol has been observed under drought conditions [39]. Nevertheless, the protective function of AsA and Vitamin E has been observed for other types of abiotic stresses, although little is known about the effects of AsA and Vitamin E on seed qualities and hormones in relation to high-temperature stresses. Brassinosteroids are steroidal plant hormones that also play an important role in alleviating the effects of high temperatures on plants. Extreme temperatures augment stress indications, i.e., necrotic areas on the leaves of bananas. However, upon the application of the trihydroxylated spirotane analog of BR, the high-temperature stress was significantly decreased in treated plants, and these plants showed improved heights compared with untreated plants [40].

Jasmonates [Methyl jasmonate+ jasmonic acid] are crucial cellular regulators that are involved in several plant developmental processes, including seed germination, callus growth, primary root growth, flowering, gum and bulb formation, and senescence [41, 42,]. Jasmonates stimulate plant defense responses to a variety of biotic and abiotic stresses [43]. In addition, the exogenous application of MeJA in A. thaliana confers basal thermo-tolerance and protection against heat shock [44]. Triazoles (Tr), as plant growth regulators, protect plants from several abiotic stresses, e.g., thermal stress and water-deficient stress [45]. The mechanism underlying the role of triazoles in stress protection involves hormonal changes, including cytokinin augmentation, increased ABA and reduced ethylene [46, 47].

Despite the significance of the milling results to worldwide food safety and the economy, there are few studies on the milling quality and content of different hormones in crop seeds, leaving a notable gap in the literature on this important issue. To fill this gap, in the present study, we used different combinations of plant growth regulators with several antioxidants (Ve, Vc, Br, MeJA, and Tr). The objectives of the present study were to (a) evaluate the response of rice grain milling quality, grain appearance quality, and grain viscosity traits to high day and high night temperature stresses and (b) characterize the influence of different plant growth regulators on rice quality under high-temperature stress.

## Materials and Methods

### Plant husbandry and growth conditions

Present studies were performed in a greenhouse at the Huazhong Agricultural University, Wuhan, China (30° 47^/^N, 114° 35^/^ E), during the 2013 and 2014 growing seasons. Two indica rice (*Oryza sativa* L.) cultivars viz., IR-64 and Huanghuazhan (HHZ), having a similar plant architecture (medium stature) but different responses to temperature, were used in the present study. HHZ is tolerant to high-temperature stress, whereas IR-64 is sensitive to high temperature. From 15 May to 25 September, rice plants were cultivated under natural conditions. To facilitate germination, a wet towel was used to maintain the seeds’ moisture for two days. Different seedling trays were used after germination, and the seeds were subsequently placed in each cell (1 seed per cell). Three weeks after sowing, three seedlings were transplanted to plastic pots (21.6 cm lower inside diameter, 27.2 cm upper inner diameter, 27.2 cm height and 0.15 cm thickness) filled with 12 kg of air-dried soil. In both years, IR-64 was sown for 12 more days than HHZ to match the heading dates of these varieties. The soil was silt loam containing sand, silt and clay at 32%, 54%, and 14%, respectively. To each pot, 10 g of compound fertilizer (16% N: 16% P: 16% K) was applied. Standard practices for pot experiments were followed, and during the experimental stage, no pest or disease dilemma was observed.

### Treatments

Three indoor controlled-environment growth chambers (Climatrons, Southeast Ningbo Instruments Ltd, Zhejiang, China) set at three different temperature treatments, i.e., HDT (high day temperature), HNT (high night temperature) and AT (ambient temperature) were provided. HDT plants were grown in 12h days (7am- 7pm) at 35°C ± 2 and 12h nights at 28°C ± 2. HNT plants received 12h days (7am- 7pm) at 28°C ± 2 and 12h nights at 32°C ± 2. While, the control (AT) plants were grown at 28°C ± 2 for both day and night (12 h-day/12 h-night cycles). The heat treatments were employed from the booting stage to physiological maturity of the plants because most of the damage to rice from high-temperature stress occurs between these durations. Throughout the experimental period, humidity was kept constant at 75%. The photosynthetic photon flux density inside the growth chamber was maintained at 1000 μM m^-2^ sec^–1^, but the CO_2_ inside the chamber was not measured. To reduce the variations, the plant pot locations of both cultivars were regularly reshuffled within a growth chamber at 15-day intervals to provide uniform environmental conditions.

Different combinations of plant growth regulators were exogenously applied three times at 30, 35, and 40 days after emergence (DAE) to enable thorough coverage prior to imposing heat stress. The different PGR treatments were (1) vitamin C + vitamin E + methyl jasmonates + brassinosteroids (Vc+Ve+MeJA+Br), (2) brassinosteroids + triazoles + methyl jasmonates (Br+Tr+MeJA), (3) vitamin C + vitamin E (Vc+Ve), (4) methyl jasmonates (MeJA), and (5) nothing applied control (NAC). Vc, Ve, MeJA, Br and Tr were applied at rates of 1.4, 6.9, 1.8, 4.0 and 0.55 ppm solution, accordingly in the respective treatments. Vc was dissolved in de-ionized water, and Ve was dissolved in a small amount of ethyl alcohol; de-ionized water was further added to bring the solution to the desired volume. Both Vc and Ve were purchased from Sigma-Aldrich, Shanghai, China and Br, MeJA, and Tr were obtained from Olchemim Ltd, Šlechtitelů, Olomouc, Czech Republic.

### Observations

#### Grain qualitative traits

After harvesting, the rice grain was stored at room temperature for three months prior to quality testing. Grain milling and appearance quality indices (brown rice, milled rice, head rice), chalkiness (PGWC, and PACE), grain length and width, and grain area were determined following the method of Chen et al. [48]. To measure these traits, the rice kernel samples were dehulled using a laboratory dehuller (SY88-TH, BRIC, Korea) (dehull rough rice into brown rice), and 10 g of brown rice was obtained as a subsample. The bran was removed using a laboratory polisher (Pearleat, Kett, Japan). Subsequently, head rice was separated from milled rice using a grain separator (HFQS-13*20, China). Approximately 100 grains were scanned to analyze the appearance quality (Epson Expression 1680 Professional, Epson, America) following the method of Yoshioka [49], with some modifications. Digital images of each head rice subsample were obtained using a scanner with a white board as background to increase the contrast between the chalky and translucent areas in the images. Subsequently, image analysis software (Image J, the National Institutes of Health, USA) was used to analyze the parameters of the subsamples, such as grain length, grain width, chalky grain percentage and chalkiness, in the digital images.

### Rapid viscoanalyzer (RVA) profile characteristics and grain amylose contents

The rapid viscoanalyzer (RVA) profile characteristics and grain amylose contents were determined. The rapid viscoanalyzer (RVA) profile reflects starch gelatinization, disintegration, swelling and gelling ability, and this information is often used to evaluate rice cooking and eating quality [50]. In this experiment, rice starch viscosity was assayed using a RVA (Model RVA-3D, Newport Scientific, Sydney, Australia) according to Han et al. [51]. The characteristics of the RVA profile were expressed as peak viscosity, trough viscosity, final viscosity, breakdown (difference between peak viscosity and trough viscosity) and setback (difference between final and peak viscosities). The viscosity was expressed in rapid visco units (RVU), with 1 RVU equaling approximately 12 centipoises.

### Statistical analysis

The experiments were arranged as a two-factor completely randomized design for two cultivars. Each treatment was replicated four times in each year. In the combined analysis of the data, the interaction year and treatments were non-significant; therefore, the data for both years were pooled and presented with the interaction of high temperature and soil fertilization treatments. The data were statistically analyzed using the Statistix software, 8.1 (Analytical Software, Tallahassee, FL, USA). The differences among treatments were separated using the least significant difference test at the 0.05 probability level.

## Results

### Rice grain milling and appearance qualities

Both the high day and high night temperature stresses applied after the booting stage of crop development negatively affected the rice grain appearance and milling quality of both cultivars (Table 1). The effect of applied PGRs were also significant (p≤ 0.05), except for grain length (GL) and grain area (GA) for both cultivars and grain width (GW) for the heat-susceptible cultivar IR-64. The interaction of heat × PGR was non-significant (p>0.05) for all grain milling attributes, except percent area of endosperm chalkiness, in the heat-tolerant cultivar HHZ (Table 1). HDT and HNT reduced the grain length, grain width, grain area and percentage of head and milled rice, whereas the percent grain with chalkiness and percent area of endosperm chalkiness were increased in both cultivars. The effects of HNT were more severe than those of HDT, resulting in a 6–21% reduction in grain appearance, 76–134% increase in endosperm chalkiness and 7–27% reduction in grain milling attributes compared with AT. The intensity of damage by HDT or HNT on grain appearance and milling attributes varied in both cultivars. IR-64 were more susceptible to heat stress for GA (-16%) and head rice % (-27%) compared with HHZ (Table 1).

**Table 1:** The effects of high temperature stress and exogenously applied plant growth regulators on the milling and appearance grain qualities of two rice cultivars (Avg. of two years).

Tem	PGR	Grain length (mm)		Grain width (mm)		Grain area (mm^2^)		Percent grains with chalkiness (%)		Percent area of chalkiness endosperm (%)		Head rice (%)		Milled rice (%)	
		IR-64	HHZ	IR-64	HHZ	IR-64	HHZ	IR-64	HHZ	IR-64	HHZ	IR-64	HHZ	IR-64	HHZ
HNT	Vc+Ve+MeJA+Br	5.7 a	5.2 a	1.99 bcd	2.01 cde	11.47 de	11.61 abc	80.81 cde	54.02 bc	21.6 efg	11.7 de	48.61 efg	60.39 c-f	66.74 bc	72.98 ab
	Br+Tr+MeJA	5.6 a	5.1 a	1.91 cd	1.92 def	11.43 e	11.18 abc	86.48 abc	58.62 ab	26.3 cd	16.6 b	43.64 hi	55.50 e-h	62.12 cd	68.25 cd
	VC+Ve	5.7 a	5.1 a	1.96 bcd	1.98 cde	11.33 de	11.43 abc	83.90 bcd	56.82 b	24.1 de	13.5 cd	46.35 fgh	58.28 d-g	64.63 c	70.51 bc
	MeJA	5.6 a	5.1 a	1.88 d	1.81 ef	11.27 e	10.97 bc	88.58 ab	62.37 ab	31.2 b	18.9 a	41.29 ij	53.16 gh	59.60 e	65.70 e
	NAC	5.6 a	5.0 a	1.87 d	1.76 f	11.11 e	10.81 c	93.58 a	66.04 a	35.0 a	20.6 a	39.22 j	50.17 h	58.29 e	64.03 e
HDT	Vc+Ve+MeJA+Br	5.9 a	5.5 a	2.12 b	2.15 bc	13.09 a-d	11.85 a	72.08 f	33.1 fgh	17.3 hij	6.6 gh	52.81 cde	63.74 bcd	70.70 a	75.62 a
	Br+Tr+MeJA	5.9 a	5.4 a	2.06 bcd	2.05 cd	12.97 b-e	11.54 abc	78.23 def	38.32 ef	22.7 ef	10.9 e	47.53 fgh	58.34 d-g	65.98 bc	71.50 bc
	VC+Ve	5.8 a	5.5 a	2.09 bc	2.11bcd	12.99 a-d	11.76 ab	74.40 ef	34.54 fg	19.8 fgh	8.6 f	50.07 def	60.76 c-f	68.95 ab	73.83 ab
	MeJA	5.7 a	5.4 a	2.01bcd	1.97 cde	12.94 cde	11.30 abc	80.15 cde	43.92 de	26.7 cd	12.6 de	45.21 ghi	56.07 e-h	63.47 c	68.95 cd
	NAC	5.7 a	5.1 a	1.97 bcd	1.96 c-f	12.86 cde	11.25 abc	85.13 bcd	46.95 cd	29.0 bc	14.7 bc	44.02 hi	54.84 fgh	61.43 cd	67.01 cd
AT	Vc+Ve+MeJA+Br	6.3 a	5.5 a	2.41a	2.72 a	13.72 a	12.03 a	45.45 h	22.14 i	12.9 k	5.0 h	62.05 a	70.01 a	72.11 a	76.19 a
	Br+Tr+MeJA	6.3 a	5.5 a	2.40 a	2.65 a	13.73 ab	11.90 a	49.93 gh	25.49 hi	15.9ijk	6.1 gh	56.73 bc	65.10 abc	66.49 bc	72.28 bc
	VC+Ve	6.3 a	5.5 a	2.41a	2.66 a	13.71 a	11.94 a	46.83gh	23.49 i	14.5 jk	5.2 gh	59.26 ab	67.ab	69.63 ab	74.11 ab
	MeJA	6.2 a	5.5 a	2.39 a	2.16 bc	13.23 ab	11.57 abc	48.28 gh	26.47 ghi	17.1 hij	7.1 fg	54.70 c	62.95 bcd	65.04 bc	70.31 bc
	NAC	6.2 a	5.4 a	2.37 a	2.27 b	13.13 abc	11.49 abc	52.93 g	28.84 ghi	18.6 ghi	8.8 f	53.53 cd	61.28 cde	63.55 c	68.78 cd
Temperature		ns	ns	**	**	**	**	**	**	**	**	**	**	**	**
PGR		ns	ns	ns	**	ns	ns	**	**	**	**	**	**	*	*
Temperature × PGR		ns	ns	ns	ns	ns	ns	ns	ns	ns	**	ns	ns	ns	ns
LSD:P<0.05 (Tem × PGR)		1.01	0.53	0.22	0.21	0.80	0.88	7.21	8.43	3.51	1.90	4.40	3.51	3.55	3.69
CV		6.73	6.77	6.80	6.73	4.50	5.37	7.13	14.30	11.17	12.6	6.23	7.06	7.49	6.63

** and * denote significance at the 0.01 and 0.05 probability level, respectively.

Within a column for each cultivar, means not sharing a common letter (a, b, c…) are significantly different at 0.05 probability level according to least significant difference (LSD). ns: non-significant, CV: Coefficient of variation, PGR: Plant growth regulators, HHZ: Huanghuazhan (heat tolerant), IR-64 (heat susceptible). HDT: high day temperature, HNT: high night temperature, AT: ambient temperature (control). Different PGRs viz., vitamin C (Vc), vitamin E (Ve), methyl jasmonates (MeJA), brassinosteroids (Br) and triazoles (Tr) were applied at the rate of 1.4, 6.9, 1.8, 4.0 and 0.55 ppm solution, respectively in respective treatments, NAC: nothing applied control.

All PGRs effectively enhanced stress tolerance in both cultivars, but the level of stress mitigation varied, depending on the PGR combination applied. The PGR combination of Vc+Ve and Vc+Ve+MeJA+Br outcompeted all other combinations under HDT and HNT. The Vc+Ve+MeJA+Br combination increased rice GW 10% under HDT and 14% under HNT stress. The grain and endosperm area under chalkiness was significantly reduced, and the percentage of head and milled rice was improved when PGRs were applied. The highest improvement in percentage of head rice (23%) was recorded for IR-64 under HNT stress after the application of Vc+Ve+MeJA+Br. Recovery from chalkiness was greater (55%) in HHZ than in IR-64 (41%). The least recovery (11–15%) was reported for milled rice percentage under HDT stress (Table 1).

### Grain viscosity and gelatinization temperature

Both the rapid visco-analyzer (RVA) profile characteristics and the gelatinization temperatures were significantly (p≤0.01) affected by high-temperature stress (Table 2). These grain attributes responded differently to HDT and HNT cycles. High-temperature stress increased the grain breakdown, set back and gelatinization temperature. The grain viscosity analysis showed a decrease in peak, trough and final viscosities, whereas the consistence viscosity was increased under high temperature stress levels (Table 2). The foliar application of PGRs was generally found to peak viscosity, break down, and trough viscosity, while decreased the consistence viscosity and set back. Statistical evaluation of the temperature and PGR interaction proposed a non-significant effect for all attributes in both cultivars (Table 2). HDT reduced the peak, trough and final viscosities by 16%, 54% and 2%, respectively, in IR-64 and by 5%, 38% and 10%, respectively, in HHZ compared with AT. The respective reductions in the peak, trough and final viscosities due to HNT were 29%, 57% and 3%, respectively, for IR-64 and 16%, 45% and 3%, respectively, for HHZ. However, both HDT and HNT improved the consistence viscosity in both cultivars. The reductions in grain viscosities were greater in IR-64 under HNT compared with their counterparts. The impact of HDT was more severe on grain break down and gelatinization temperature, whereas HNT increased grain set back (Table 2).

**Table 2:** The effects of high temperature stress and exogenously applied plant growth regulators on Rapid viscoanalyzer (RVA) profile characteristics of two rice cultivars (Avg. of two years).

Tem	PGR	Peak viscosity		Break down		Trough viscosity		Final viscosity		Set back		Consistence viscosity		Gelatinization temperature (°C)	
		Rapid visco units.													
		IR-64	HHZ	IR-64	HHZ	IR-64	HHZ	IR-64	HHZ	IR-64	HHZ	IR-64	HHZ	IR-64	HHZ
HNT	Vc+Ve+MeJA+Br	191.4 de	253.8 cde	64.8 g	81.2 f	126.6 bcd	172.6 efg	227.6 a	266.9 a-e	36.2 cde	13.1 ef	101.0 de	94.3 e	77.2 ab	74.9 abc
	Br+Tr+MeJA	177.1 efg	233.4 efg	73.7 ef	89.0 de	103.3 d-g	144.4 hi	220.5 a	258.7 cde	43.4 abc	25.3 c	117.1 bc	114.4 c	79.8 a	76.3 ab
	VC+Ve	186.5 def	246.0 def	68.8 fg	84.9 ef	117.7 cde	161.0 fgh	226.1a	266.3 a-e	39.5 bcd	20.3 d	108.4 cde	105.2 d	78.6 ab	75.2 abc
	MeJA	167.6 fg	225.1 fg	77.9 de	93.1 cd	89.7 fgh	132.0 i	214.4 a	254.0 c-f	46.8 ab	29.0 b	124.7 ab	122.1 b	80.9 a-d	76.9 a
	NAC	159.7 g	218.2 g	81.2 cd	96.0 c	78.5 h	122.1 i	209.8 a	251.2 def	50.0 a	33.1 a	131.2 a	129.1 a	77.2 a-d	77.0 a
HDT	Vc+Ve+MeJA+Br	221.9 abc	288.2 ab	77.9 de	92.6 cd	144.0 b	195.5 de	232.6 a	291.3 a	10.7 h	3.1 h	88.6 f	95.8 e	81.6 a-d	73.9 bc
	Br+Tr+MeJA	202.0 cd	266.5 bcd	87.7 bc	103.7 b	114.2 c-f	162.8 fgh	224.7 a	277.4 abc	22.8 gh	10.8 fg	110.5 cd	114.5 c	76.3 abc	75.0 abc
	VC+Ve	214.2 bc	277.9 abc	83.0 cd	97.7 c	131.2 bc	180.2 ef	230.8 a	286.0 ab	16.6 fg	8.1 g	99.6 e	105.8 d	78.4 b-f	74.3 abc
	MeJA	188.5 def	256.6 cde	93.5 ab	107.9 ab	95.0 e-h	148.6 ghi	218.8 a	272.5 a-d	30.3 ef	16.0 e	123.8 ab	123.9 b	77.4 def	75.5 abc
	NAC	180.8 d-g	247.0 def	96.5 a	110.5 a	84.3 gh	136.5 hi	211.9 a	269.8 a-e	31.2 def	22.8 cd	127.6 a	133.3 a	79.9 c-f	75.7 abc
AT	Vc+Ve+MeJA+Br	240.8 a	293.8 a	34.7 h	30.7 i	206.1 a	263.1 a	221.1 a	267.2 a-e	-19.7 k	-26.6 k	15.0 i	4.1 i	74.3 ef	73.2 c
	Br+Tr+MeJA	233.1 ab	254.0 cde	38.0 h	34.0 ghi	195.0 a	219.9 cd	222.2 a	232.3 f	-10.9 ij	-21.7 j	27.1 gh	12.3 h	74.7 def	73.4 c
	VC+Ve	237.6 a	285.5 ab	36.7 h	32.2 hi	200.9 a	253.2 ab	219.7 a	259.9 b-e	-17.9 jk	-25.5 k	18.8 hi	6.7 i	74.7 f	73.4 c
	MeJA	228.4 ab	268.0 bcd	40.0 h	36.7 gh	188.4 a	231.3 bc	218.8 a	248.6 def	-9.6 ij	-19.4 j	30.4 g	17.3 g	74.8 a-d	73.8 bc
	NAC	223.9 abc	259.7 cd	40.8 h	38.1 g	183.1 a	221.6 cd	216.9 a	244.3 ef	-7.0 i	-15.4 i	33.8 g	22.7 f	75.5 a-e	73.9 bc
Temperature		**	**	**	**	**	**	**	**	**	**	**	**	**	**
PGR		**	**	**	**	**	**	**	**	**	**	**	*	ns	**
Temperature × PGR		ns	ns	ns	ns	ns	ns	ns	ns	ns	ns	ns	ns	ns	ns
LSD:P<0.05 (Tem × PGR)		22.32	24.26	6.81	5.59	24.10	27.93	29.16	26.06	8.65	3.56	10.37	4.73	3.2	2.74
CV		7.70	6.60	7.21	5.22	12.65	10.72	9.26	6.95	34.47	51.5	8.68	4.51	6.9	5.58

** and * denote significance at the 0.01 and 0.05 probability level, respectively.

Within a column for each cultivar, means not sharing a common letter (a, b, c…) are significantly different at 0.05 probability level according to least significant difference (LSD). ns: non-significant, CV: Coefficient of variation, PGR: Plant growth regulators, HHZ: Huanghuazhan (heat tolerant), IR-64 (heat susceptible). HDT: high day temperature, HNT: high night temperature, AT: ambient temperature (control). Different PGRs viz., vitamin C (Vc), vitamin E (Ve), methyl jasmonates (MeJA), brassinosteroids (Br) and triazoles (Tr) were applied at the rate of 1.4, 6.9, 1.8, 4.0 and 0.55 ppm solution, respectively in respective treatments, NAC: nothing applied control.

A significant improvement in grain viscosity and breakdown was achieved by the foliar application of PGRs. Cultivar IR-64 was more responsive to PGRs and higher increases in grain viscosity attributes, except for set back, were recorded for this cultivar. The PGR combination Vc+Ve+MeJA+Br showed maximum improvement in these attributes, however, this combination was statistically similar to Vc+Ve. The PGR combination Br+Tr+MeJA and MeJA alone were least effective (Table 2).

## Discussion

Grain appearance and milling qualities were severely affected by high-temperature stress and PGR application in both rice cultivars. The effect of HNT was more severe compared with HDT stress. Few reports on the impact of HNT on rice grain quality and phytochrome concentration have been published. Recently, Lyman et al. [52] reported up to 10% reduction in rice grain yield resulting from increasing temperatures in South and Southeast Asia. This reduction was low compared with the ongoing heat stress pot trials, showing a grain yield reduction of 43% for HDT and 72% for HNT after the booting stage (data not shown). A higher rate of grain filling up to 40% and shorter filling period have been reported [53] as major causes of grain quality damage. Under heat stress, annual plants attempt to complete their life cycle as soon as possible, resulting in a hormonal imbalance that activates functional and structural changes during grain formation. Some of the reported grain appearance changes are the percentage of brown rice, milled rice, head rice, imperfect rice, chalky grain and endosperm chalkiness [21]. Grains with opaque spots were characterized as chalky [49]. This spots downgrade rice quality but disappear upon cooking and do not affect taste or aroma. The development of numerous air spaces between loosely packed starch granules is a major cause for chalky appearance, resulting in changes in light reflection [54]. Grains with chalkiness depicted higher levels of long chains of amylopectin accumulation, which is considered a major reason for the development of grain chalkiness. Umemoto and Terashima [55] confirmed a significant reduction in grain weight and amylose content in chalky grains for Japonica cultivars under heat stress. The rice milling quality and recovery for grain dimensions were also highly dependent on the level of temperature stress and cultivars [22. 23]. Zhu et al. [56] reported that the grain length, width and amylose content were decreased under heat stress, whereas grain and endosperm chalkiness and protein contents were increased. These authors further elaborated that increased chalkiness might reflect reduced photo-assimilate partitioning and translocation to grain. Chalky kernels break easily during processing, thereby decreasing the head rice yield during milling [57]. Exposure of HNT during grain filling stage altered the enzymatic activity [18, 24], leading to irregular packing of starch granules resulting in the increased chalkiness [25]. Recently, Shi et al. [26] reported that HNT reduced in head rice yield and grain width, altered the amylose content, while increased the increased the chalkiness in various studied genotypes.

The results of the present study revealed that rice grain rheological properties (peak, trough and final viscosity) were decreased, whereas consistence viscosity, breakdown, set back and gelatinization temperature were increased under heat stress. The difference between the final and peak viscosity was referred to as set back and is considered a grain starch quality indicator. Starch exhibits unique viscosity behavior with changes in temperature and concentration. Han et al. [51] reported that higher peak viscosity and lower trough viscosity are associated with better-tasting rice. Rice grain quality (cooking and sensory properties) is strongly correlated with grain rheological properties, and these properties are affected by the accumulation and deposition of starch [58]. Not only is inferior grain quality under heat stress is regulated by starch content, but changes in the accumulation of starch-related proteins also play a vital role by impeding the normal metabolic pathways and inhibiting starch deposition [59]. Cooper et al. [18] showed higher lipid contents in rice grains under elevated temperature stress. Lipid bodies are primarily present in the aleurone layer of seeds and have been confirmed in the endosperm layer as being cross linked with starch granules. These cross linked molecules influence the viscoelastic properties by forming an inclusion complex with amylose, which controls the swelling capacity of starch granules in kernels [60].

The plant growth regulators Vc, Ve, MeJA, Br and Tr can significantly mitigate heat stress by ameliorating the ill effects on rice grain appearance, milling and quality aspects. Improved grain viscosity was also associated with the exogenous foliar application of PGR combinations. PGR combinations decreased grain breakdown, set back and gelatinization temperature, thus indicating a positive role for these factors in heat stress.

## Conclusions

In conclusion, high-temperature stress, particularly HNT, severely diminished the grain appearance quality, milling quality and viscosity traits in both rice cultivars. High temperatures reduced the grain length, grain width, grain area, head rice percentage and milled rice percentage and the increased chalkiness percentage and percent area of endosperm chalkiness in rice. Nevertheless, exogenously applied PGRs were effective in alleviating the detrimental effects of HDT and HNT stresses. The combination of Vc+Ve+MeJA+Br remained superior to all other PGR treatments for most of the studied characteristics.
